The article "Photo-responsive hole formation in the monolayer membrane wall of a supramolecular nanotube for quick recovery of encapsulated protein" was retracted in 2024. Reasons: fabricated or falsified images; an official misconduct investigation; misconduct by an author; errors in the images.

# Photo-responsive hole formation in the monolayer membrane wall of a supramolecular nanotube for quick recovery of encapsulated protein†

**DOI:** 10.1039/d2na00035k

**Published:** 2022-02-28

**Authors:** N. Kameta, Y. Kikkawa, Y. Norikane

**Affiliations:** Nanomaterials Research Institute, Department of Materials and Chemistry, National Institute of Advanced Industrial Science and Technology (AIST) Tsukuba Central 5, 1-1-1 Higashi Tsukuba Ibaraki 305-8565 Japan n-kameta@aist.go.jp +81-29-861-4545 +81-29-861-4478; Research Institute for Advanced Electronics and Photonics, Department of Electronics and Manufacturing, AIST Tsukuba Central 5, 1-1-1 Higashi Tsukuba Ibaraki 305-8565 Japan

## Abstract

Nanotubes with a single monolayer membrane wall comprised of a synthetic glycolipid and one of two synthetic azobenzene derivatives were assembled. X-ray diffraction, infrared, UV-visible, and circular dichroism spectroscopy clarified the embedding style of the azobenzene derivatives in the membrane wall, revealing that, depending on their different intermolecular hydrogen bond strengths, one azobenzene derivative was individually dispersed whereas the other formed a *J*-type aggregate. The non-aggregated derivative was insensitive to UV irradiation due to tight fixation by the surrounding glycolipid. In contrast, the aggregated derivative was sensitive to UV irradiation, which induced *trans*-to-*cis* isomerization of the derivative and disassembly of the *J*-type aggregate. Subsequent dissociation of the derivative into the bulk solution resulted in the formation of many nanometer-scale holes in the membrane wall. Although a model protein encapsulated within the nanotubes was slowly released over time from the two open ends of the nanotubes without UV irradiation, exposure to UV irradiation resulted in faster, preferential release of the protein through the holes in the membrane wall. The present findings are expected to facilitate the development not only of efficient means of recovering guest compounds stored within nanotubes but also the development of novel stimuli-responsive capsules in biological and medical fields.

## Abstract 2

Photoisomerization of an azobenzene derivative embedded in the glycolipid monolayer membrane wall of a nanotube resulted in the formation of many holes in the membrane wall for release of an encapsulated protein.

## Introduction

Supramolecular nanotubes formed by assembly of organic molecules such as lipids possess a one-dimensional cavity with a tunable diameter and chemically functionalizable surface.^1^ Because of their high aspect ratios (length/diameter > 100–100 000), these cavities can be used as containers for the slow or sustained release of drugs, channels for the transport or separation of biomolecules, and templates for the production of conformationally controlled polymers and inorganic nanorods.^2^ The confinement effect of the nanotube cavity is also useful for stabilizing proteins or accelerating their refolding.^2^ However, the length of the nanotube cavity often hinders the recovery of encapsulated compounds. Indeed, compared with recovery from spherical nanocapsules or nanorings (very short nanotubes), recovery from nanotubes takes much longer and the process is much less efficient.^3^ To address this issue, methods to decompose or transform nanotubes to rapidly release encapsulated compounds have been proposed, and there are many reports describing supramolecular nanotubes that are decomposed or transformed in response to various stimuli such as pH,^4^ salts,^5^ metal ions,^6^ additives,^7^ solvents,^8^ dilution,^9^ temperature,^10^ light,^11^ ultrasound,^12^ and electric potential.^13^ However, there is little information available on the actual recovery of the encapsulated compounds from such stimuli-responsive nanotubes.

The article "Photo-responsive hole formation in the monolayer membrane wall of a supramolecular nanotube for quick recovery of encapsulated protein" was retracted in 2024. Reasons: fabricated or falsified images; an official misconduct investigation; misconduct by an author; errors in the images.

Many of the stimuli that can be used to decompose or transform supramolecular nanotubes can also denature proteins. Therefore, for supramolecular nanotubes that are to encapsulate proteins, a means of releasing the encapsulated protein without affecting the protein structure is needed. Of the various stimuli that have been reported to date, photoirradiation is the safest in this regard. Previously, we reported self-assembling photo-responsive nanotubes constructed from amphiphilic molecules modified with an azobenzene unit or a nitrobenzyl group.^14^ Upon photoirradiation of these nanotubes, the diameter of the cavity shrank from 18–20 nm to <1–2 nm as a result of *trans*-to-*cis* photoisomerization of the azobenzene unit or photochemical cleavage of the nitrobenzyl group, with these transformations leading to the release of encapsulated proteins and DNA into the bulk solution.^15^ However, because the final diameter of the cavity (1–2 nm) was smaller than the sizes of the proteins (3–4 nm) and the width of duplex DNA (2 nm), the squeezing that occurred due to the shrinking of the nanotube resulted in marked changes to the native structures of the proteins and the duplex formation of the DNA. Thus, an alternative means of achieving the rapid release of proteins from nanotubes that does not negatively impact the protein structure is needed.

Here, we constructed a photo-responsive nanotube consisting of a glycolipid monolayer membrane in which aggregates of an azobenzene derivative were embedded. Photoirradiation of the nanotube led to *trans*-to-*cis* isomerization and subsequent dissociation of the azobenzene derivative from the nanotube, which in turn resulted in the formation of many nanometer-scale holes in the membrane wall. These holes then acted as channels for the rapid release of an encapsulated protein into the bulk solution, with the rate of release *via* the holes in the membrane wall being much faster than that from the two original open ends of the nanotube.

The article "Photo-responsive hole formation in the monolayer membrane wall of a supramolecular nanotube for quick recovery of encapsulated protein" was retracted in 2024. Reasons: fabricated or falsified images; an official misconduct investigation; misconduct by an author; errors in the images.

## Experimental

### Morphological observations

Aqueous dispersions of nanostructures were dropped onto carbon grids, and the grids were stored in a vacuum desiccator for 24 h. To clearly visualize the nanotube channels, an aqueous solution of phosphotungstate (2 wt%) was dropped onto the individual grids as a negative staining reagent. The grids were observed under a scanning electron microscope (S-4800, Hitachi) at 10 kV. The transmission mode was operated at 30 kV.

### Structural analysis

Lyophilized nanostructures were analyzed with a Rigaku diffractometer (Type 4037) using graded *d*-space elliptical side-by-side multilayer optics, monochromatic Cu KR radiation (40 kV, 30 mA), and an imaging plate (R-Axis IV). The exposure time was 5 min with a 150 mm camera length. The lyophilized nanostructures were also analyzed with a Fourier transform infrared spectrometer (FT-620, JASCO) operated at 4 cm^−1^ resolution and equipped with an unpolarized beam, an attenuated total reflection accessory system (Diamond MIRacle, horizontal attenuated total reflection accessory with a diamond crystal prism, PIKE Technologies), and a mercury cadmium telluride detector. Variable temperature infrared spectra were measured by attaching an infrared microscope (MICRO-20, JASCO) and a Mettler FP82 hot stage (linked to a Mettler FP90 with an accuracy of 0.4 °C) to the spectrometer. Absorption and circular dichroism spectra of the nanostructures dispersed in water were measured with a UV-Vis spectrophotometer (U-3300, Hitachi) equipped with a temperature control unit (BU150A, YAMATO) and a spectropolarimeter (J-820, JASCO) equipped with a temperature control unit (PTC-423L, JASCO). The lyophilized nanostructures (1 mg) and water (20 μL) were placed in an aluminum pan for thermal analysis with a differential scanning calorimeter (DSC 6100, SEIKO) equipped with a nitrogen gas cooling unit.

### Photoisomerization reaction

A super-high-pressure mercury lamp (500 W) with appropriate filters was used for UV irradiation of aqueous dispersions of nanostructures. The test solutions were placed in quartz cells (length, 1 mm). The *trans*-to-*cis* isomerization of azobenzene components in the nanostructures upon UV irradiation at 365 nm was monitored with a UV-Vis spectrophotometer (UV-3150, Shimadzu).

The article "Photo-responsive hole formation in the monolayer membrane wall of a supramolecular nanotube for quick recovery of encapsulated protein" was retracted in 2024. Reasons: fabricated or falsified images; an official misconduct investigation; misconduct by an author; errors in the images.

### Encapsulation and release of GFP

An aqueous solution (1 mL) of GFP (Clontech, Recombinant GFP protein, 50 μg, in 10 mM Tris–HCl at pH 8.0) was mixed with lyophilized nanotubes (5 mg). After aging overnight, the aqueous dispersion was filtered through a polycarbonate membrane with a pore size of 0.2 μm (MILLIPORE). The residual nanotubes were washed several times to remove GFP from the outside of the nanotubes. To calculate the amount of GFP encapsulated in the nanotubes, the nanotubes were completely decomposed by addition of 5% Triton X-100. The amount of GFP released from the nanotubes was calculated to be 4.5–4.8 μg by using a fluorescence spectrophotometer (F-4500, Hitachi) with the excitation and emission wavelengths set at 472 nm and 509 nm, respectively. The recovery ratio of GFP was quantitatively determined by using a BCA protein assay kit (Pierce).

For evaluation of the time-dependent release ratio of GFP, nanotubes encapsulating GFP were stored in water at pH 6.8. After a certain time with or without UV irradiation, the aqueous dispersion was subjected to membrane filtration. The amounts of GFP released into the filtrate and GFP remaining in the nanotubes corrected as the residue were estimated by fluorescence microscopy as described above. The amount of azobenzene derivative dissociated from the nanotubes *via* photoisomerization was estimated by UV-Vis spectroscopy.

### Fluorescence microscopy

Nanotubes encapsulating GFP were stored on glass plates. After dropping water onto the nanotubes, each glass plate was subjected to UV irradiation for 5 min. GFP encapsulated in the nanotubes and GFP released from the nanotubes were monitored by using an inverted microscope (IX71, Olympus) equipped with a CCD camera (ORCA-ER, Hamamatsu). The excitation optical source comprised a high-pressure mercury lamp (100 W, BH2-REL-T3, Olympus) and a 470–495 nm band-pass filter. The fluorescence microscopic images were recorded on a personal computer by using the Aquacosmos system (Hamamatsu).

## Results and discussion

### Nanotube construction by co-assembly of a glycolipid and an azobenzene derivative

Previously, we reported a synthetic glycolipid comprising an oligomethylene spacer with a glucose headgroup at one end and a carboxyl headgroup at the other (GlcC_18_, Fig. 1) that self-assembled in water to form a nanotube (GlcC_18_-tube).^16^ Each GlcC_18_-tube consisted of five to seven stacked monolayer membranes in which the GlcC_18_ was packed in parallel fashion. In the present study, with the goal of introducing photo-responsiveness to GlcC_18_-tube, we designed and synthesized two azobenzene derivatives each also with a glucose headgroup (GlcAzo and GlcGlyAzo; Fig. 1 and S1–S4, ESI†).

The article "Photo-responsive hole formation in the monolayer membrane wall of a supramolecular nanotube for quick recovery of encapsulated protein" was retracted in 2024. Reasons: fabricated or falsified images; an official misconduct investigation; misconduct by an author; errors in the images.

**Fig. 1:** Chemical structures of the glycolipid (GlcC_18_) and azobenzene derivatives (GlcAzo and GlcGlyAzo) used in the present study.

By using GlcC_18_ and the azobenzene derivatives, two novel nanotubes were generated as binary assemblies as follows. First, a film of GlcC_18_ (3.9 mg, 7.7 μmol) was prepared by evaporation of the ethanol solution. Then, GlcAzo (0.89 mg, 2.3 μmol) or GlcGlyAzo (1.0 mg, 2.3 μmol) dispersed in deionized water (1 mL) by refluxing for 10 min was poured onto the GlcC_18_ film and allowed to cool to room temperature. Scanning transmission electron microscopy analysis of the binary assemblies revealed that nanotubes were the only nanostructures produced (Fig. S5, ESI†). Reflux and subsequent cooling of GlcAzo (0.89 mg, 2.3 μmol) or GlcGlyAzo (1.0 mg, 2.3 μmol) dispersed in deionized water (1 mL) in the absence of GlcC_18_ afforded sheet-like (GlcAzo-sheet) and tape-like (GlcGlyAzo-tape) nanostructures, respectively (Fig. 2a and b). However, no such nanostructures were observed in the scanning transmission electron microscopy images of the nanotubes (Fig. S5, ESI†), indicating that GlcAzo and GlcGlyAzo were incorporated into GlcC_18_-tube. Further examination of GlcC_18_-tube containing GlcAzo or GlcGlyAzo (hereafter GlcC_18_-GlcAzo-tube or GlcC_18_-GlcGlyAzo-tube) revealed that the nanotubes had inherited the inner diameter size of GlcC_18_-tube (19–21 nm; Fig. 2c, d and e). Furthermore, the thicknesses of the walls of GlcC_18_-GlcAzo-tube and GlcC_18_-GlcGlyAzo-tube were much thinner (3–4 nm) than that of GlcC_18_-tube (15–22 nm). Because the wall thickness of GlcC_18_-GlcAzo-tube and GlcC_18_-GlcGlyAzo-tube was comparable to the molecular length of GlcC_18_ (*L* = 3.38 nm), we concluded that both types of nanotube comprised a single monolayer membrane of GlcC_18_ interspersed with GlcAzo or GlcGlyAzo. In our previous work,^17^ we reported that the molecular packing of GlcC_18_ is more disordered in the outer monolayer membranes of GlcC_18_-tube. Incorporation of GlcAzo or GlcGlyAzo can promote the disordering of the molecular packing of GlcC_18_ and disrupt the stacking of the monolayer membranes.

**Fig. 2:** (a–e) Scanning transmission electron micrographs of the indicated nanostructures. The nanochannels of (c) GlcC_18_-tube, (d) GlcC_18_-GlcAzo-tube and (e) GlcC_18_-GlcGlyAzo-tube were visualized by means of negative staining with 2 wt% phosphotungstate.

Powder X-ray diffraction (XRD) spectroscopy analysis provided further evidence that GlcC_18_-GlcAzo-tube and GlcC_18_-GlcGlyAzo-tube were formed from a single monolayer membrane (Fig. 3). In the XRD pattern of GlcC_18_-tube, a single diffraction peak in the small-angle region reflecting a stacking periodicity of the monolayer membrane (*d* spacing) of 3.02 nm was observed. However, in the XRD patterns of GlcC_18_-GlcAzo-tube and GlcC_18_-GlcGlyAzo-tube, the intensity of the peak corresponding to the *d* spacing was significantly weaker, indicating thinner walls and the absence of stacking within the monolayer membrane. The XRD patterns of GlcC_18_-GlcAzo-tube and GlcC_18_-GlcGlyAzo-tube also showed no peaks corresponding to the *d* spacings of the stacking periodicities of the bilayer membranes in GlcAzo-sheet and GlcGlyAzo-tape (*d* = 2.74 and 3.56 nm, respectively), indicating that incorporation of the azobenzene derivatives into GlcC_18_-tube occurred in preference to assembly of the derivatives into a sheet or tape. This preferential incorporation of the azobenzene derivatives occurred when a molar ratio of 10 : 3 (GlcC_18_ : GlcAzo) was used; however, when a higher molar ratio of 10 : 2 was used, the amounts of the derivatives were too low to produce only GlcC_18_-GlcAzo-tube or GlcC_18_-GlcGlyAzo-tube and GlcC_18_-tube was also formed, and when a lower molar ratio of 10 : 5 was used, excess derivative that was not incorporated into GlcC_18_-tube formed GlcAzo-sheet or GlcGlyAzo-tape (Fig. S6, ESI†).

The article "Photo-responsive hole formation in the monolayer membrane wall of a supramolecular nanotube for quick recovery of encapsulated protein" was retracted in 2024. Reasons: fabricated or falsified images; an official misconduct investigation; misconduct by an author; errors in the images.

**Fig. 3:** Left: Schematic representations of the molecular packings of the indicated nanostructures. Middle: Powder X-ray diffraction patterns of the indicated nanostructures. The *d* values indicate the stacking periodicity of the monolayer or bilayer membrane. Right: Absorption and circular dichroism spectra of aqueous dispersions of the indicated nanostructures at 25 °C (solid lines) and 90 °C (dotted lines). [GlcC_18_] = 7.7 × 10^−4^ M; [GlcAzo] = [GlcGlyAzo] = 2.3 × 10^−4^ M. *λ*_max_, absorption maximum wavelength.

The common hydrogen bonding units in GlcC_18_, GlcAzo and GlcGlyAzo, *i.e.*, the glucose headgroup^18^ and the amide group,^19^ were found to play important roles in the formation of the nanotubes. The infrared (IR) spectra of GlcC_18_-GlcAzo-tube and GlcC_18_-GlcGlyAzo-tube showed bands attributable to O–H stretching of the glucose headgroup and C=O stretching of the amide group, which were groups found to participate in the formation of the intermolecular hydrogen bond networks in the three types of nanotube (Fig. S7, ESI†). Our findings also indicate that the azobenzene derivatives in the nanotubes were oriented with the glucose headgroup at the outer surface of the monolayer membrane as a result of hydrogen bond interactions with the GlcC_18_ component (Fig. 3 and S7, ESI†).

The article "Photo-responsive hole formation in the monolayer membrane wall of a supramolecular nanotube for quick recovery of encapsulated protein" was retracted in 2024. Reasons: fabricated or falsified images; an official misconduct investigation; misconduct by an author; errors in the images.

### Spectroscopic analysis of the embedding styles of the azobenzene derivatives in the monolayer membrane

Ultraviolet-visible (UV-Vis) absorption, circular dichroism (CD) and IR spectroscopic analyses were conducted to examine how the azobenzene derivatives were embedded in the single monolayer membrane of the nanotubes (Fig. 3). The absorption maximum wavelength of the GlcAzo component of GlcC_18_-GlcAzo-tube dispersed in water at 25 °C (*λ*_max_ = 335 nm) was comparable with that of free GlcAzo dispersed in water after decomposition of the nanotube at 90 °C (*λ*_max_ = 334 nm), indicating that the GlcAzo component was individually embedded in the monolayer membrane wall. In contrast, the absorption maximum wavelength of the GlcGlyAzo component of GlcC_18_-GlcGlyAzo-tube dispersed in water at 25 °C (*λ*_max_ = 353 nm) was red-shifted compared with that of free GlcGlyAzo dispersed in water after decomposition of the nanotube at 90 °C (*λ*_max_ = 330 nm), indicating that the GlcGlyAzo component existed as a *J*-type aggregate^20^ in the monolayer membrane wall.

Such a difference in embedding style can be ascribed to the difference in the self-association ability of the GlcAzo and GlcGlyAzo components. We evaluated this self-association ability by determining the strengths of the intermolecular π–π interactions and intermolecular hydrogen bonds formed among the GlcAzo components in the GlcAzo-sheet and the GlcGlyAzo components in the GlcGlyAzo-tape. Both components formed *H*-type aggregates^21^ in their sheet and tape nanostructures, and their absorption bands were blue-shifted relative to the bands of the corresponding free components (Fig. 3). Since the degree of the blue shift in the spectrum of the GlcAzo-sheet (*λ*_max_ = 315 ← 334 nm) was similar to that in the spectrum of the GlcGlyAzo-tape (*λ*_max_ = 309 ← 330 nm), the intermolecular π–π interaction strength among the GlcAzo components was comparable with that among the GlcGlyAzo components. However, when the frequencies of the amide-I IR bands (the C=O stretching IR bands) were used as an index of intermolecular hydrogen bond strength, the wavenumber of the peak of the amide-I IR band for GlcAzo-sheet (1684 cm^−1^) was found to be higher than those of the peaks of the GlcGlyAzo-tape (1675 and 1632 cm^−1^), indicating that the intermolecular hydrogen bond strength of the GlcAzo component was weaker than that of the GlcGlyAzo component (Fig. S8, ESI†). This difference was attributed to the presence of the glycine moiety in GlcGlyAzo, which is a moiety that can form hydrogen bonds.^22^ Thus, the GlcGlyAzo component was found to be superior to the GlcAzo component in terms of self-association ability, which resulted in the GlcGlyAzo component, but not the GlcAzo component, forming *J*-type aggregates in the membrane wall of the nanotube.

The article "Photo-responsive hole formation in the monolayer membrane wall of a supramolecular nanotube for quick recovery of encapsulated protein" was retracted in 2024. Reasons: fabricated or falsified images; an official misconduct investigation; misconduct by an author; errors in the images.

Assembly and aggregation of chiral components is known to result in amplified chirality.^23^ Except for GlcC_18_-GlcAzo-tube, a split-type induced CD with negative/positive Cotton effects was observed in the absorption regions of the azobenzene derivatives, which both bore a d-glucose headgroup as a chiral source, further indicating that the azobenzene derivatives formed aggregates in GlcC_18_-GlcGlyAzo-tube, GlcAzo-sheet and GlcGlyAzo-tape (Fig. 3). The induced CD intensity of the *J*-type aggregate of GlcGlyAzo in GlcC_18_-GlcGlyAzo-tube was larger than those of the *H*-type aggregates of GlcAzo in GlcAzo-sheet and of GlcGlyAzo in GlcGlyAzo-tape. This result is reasonable considering the larger contribution of chiral packing in the formation of the tubular monolayer membrane compared with that in the formation of the planar sheet and tape morphologies.^24^

Variable-temperature IR spectroscopy revealed that the thermal phase transition of the oligomethylene spacer of the GlcC_18_ component in the nanotubes was strongly influenced by the embedded azobenzene derivatives. The CH_2_ stretching IR band (*ν*_s_(CH_2_)) is sensitive to the gel-to-liquid crystalline phase transition within membranes.^25^ A peak shift of *ν*_s_(CH_2_) to a higher frequency indicates an increase in the *gauche*/*trans* conformation ratio in the oligomethylene spacer upon heating.^26^ The thermal phase transition temperature (*T*_g-l_) of GlcC_18_-GlcAzo-tube (178 °C) was lower than that of GlcC_18_-tube (201 °C) (Fig. 4), indicating that the embedded GlcAzo component, which was individually dispersed in the monolayer membrane, caused disorder of the molecular packing of the GlcC_18_ component. In contrast, the GlcC_18_-GlcGlyAzo-tube possessed two *T*_g-l_ at 125 and 196 °C. Since the higher *T*_g-l_ was comparable with that of GlcC_18_-tube, it corresponds to the thermal phase transition of oligomethylene spacer located far from the aggregated GlcGlyAzo component in the monolayer membrane. The thermal phase transition for the lower *T*_g-l_ corresponds to the oligomethylene spacer in direct contact with the aggregated GlcGlyAzo component.

**Fig. 4:** Temperature dependence of the *ν*_s_(CH_2_) infrared band peak position of the indicated nanotubes. Each temperature as shown in red characters corresponded to the thermal phase transition temperature of the oligomethylene spacer of the GlcC_18_ component in the indicated nanotubes.

### Photoisomerization of embedded azobenzene derivatives

For GlcC_18_-GlcGlyAzo-tube dispersed in water, UV irradiation at 365 nm induced a decrease in the π–π* band (*λ*_max_ = 353 nm) of the *trans*-GlcGlyAzo component and the appearance of the π–π* (*λ*_max_ = 256 nm) and n–π* (*λ*_max_ = 430 nm) bands of the *cis* isomer (Fig. 5b).^27^ This spectral change attributed to *trans*-to-*cis* isomerization was attained within 5 min of the start of UV irradiation, even though the GlcGlyAzo component was embedded in the solid (crystalline) state monolayer membrane. Such photoisomerization was observed also in the GlcAzo-sheet and the GlcGlyAzo-tape (Fig. S9, ESI†), indicating that the photoisomerization was the result of the azobenzene derivatives being next to one another, although the photoisomerization rates of the GlcAzo and GlcGlyAzo components existing as *H*-type aggregates in the sheet and tape were slightly slower than those of the GlcGlyAzo component existing as a *J*-type aggregate in GlcC_18_-GlcGlyAzo-tube. In contrast, the absorption spectrum of GlcC_18_-GlcAzo-tube, in which the GlcAzo component was embedded in the monolayer membrane without aggregation, did not change upon UV irradiation (Fig. 5a). We ascribe this lack of photoisomerization to tight fixation of the GlcAzo component by the surrounding GlcC_18_ component. The evidence for this comes from the more stable molecular packing of GlcC_18_ component in GlcC_18_-GlcAzo-tube compared with that in GlcC_18_-GlcGlyAzo-tube, as shown by the *T*_g-l_ values of the thermal phase transition of the oligomethylene spacer of the GlcC_18_ component (see previous section).

The article "Photo-responsive hole formation in the monolayer membrane wall of a supramolecular nanotube for quick recovery of encapsulated protein" was retracted in 2024. Reasons: fabricated or falsified images; an official misconduct investigation; misconduct by an author; errors in the images.

**Fig. 5:** (a and b) Changes in absorption spectra upon ultraviolet irradiation of the indicated nanotubes dispersed in water. The red and blue spectra were recorded before ultraviolet irradiation and after ultraviolet irradiation for 5 min, respectively. Insets show the relationship between absorbance at the maximum wavelength and ultraviolet irradiation time. [GlcC_18_] = 7.7 × 10^−4^ M; [GlcAzo] = [GlcGlyAzo] = 2.3 × 10^−4^ M.

### Photoisomerization induced hole formation in the membrane wall of nanotubes

The *trans*-to-*cis* isomerization of GlcGlyAzo component of GlcC_18_-GlcGlyAzo-tube dispersed in water upon UV irradiation for 5 min led to the formation of holes in the monolayer membrane wall. Scanning electron microscopic observation revealed that the holes were oval-shaped with a wide range of diameters (13–74 nm) and were clearly distinct from the original circular holes of uniform diameter (19–21 nm) at the open ends of the tubes (Fig. 6a–c). GlcC_18_-GlcGlyAzo-tube should also have many smaller holes (<10 nm in diameters), which are difficult to be observed due to the resolution of the scanning electron microscopy in the present study. Scanning transmission electron microscopic observation and IR spectroscopic measurements clearly confirmed that the hole formation upon UV irradiation never influences not only the basic tubular morphology such as the inner diameter size and the wall thickness but also the molecular packing of GlcC_18_ within the single monolayer membrane (Fig. S10 and S11, ESI†). However, differential scanning calorimetry measurements revealed that the thermal stability of GlcC_18_-GlcGlyAzo-tube in water remarkably decreases after the hole formation (Fig. S12, ESI†). After UV irradiation of an aqueous dispersion of the nanotube for a certain time, the nanotube was passed through a polycarbonate membrane filter with a pore size of 0.2 μm, leading to the filter capturing the nanotube while the GlcGlyAzo component dissociated from the nanotube passed through into the filtrate. The time dependency of the recovery (release) ratio of the GlcGlyAzo component (Fig. S13, ESI†) indicated that dissociation of the GlcGlyAzo component from the nanotube accompanied the photoisomerization (Fig. 6d). The *cis* isomer of azobenzene has a higher polarity and solubility in water compared with those of the *trans* isomer;^28^ therefore, it is reasonable that the *cis* isomer of the GlcGlyAzo component would dissociate from the nanotube and enter the aqueous bulk solution. This indicates that the holes that formed in the monolayer membrane were the places where the GlcGlyAzo component was present as the *J*-type aggregate before UV irradiation. The variation in the shape and size of the holes is likely related to the variation in the shape and size of the *J*-type aggregate in the monolayer membrane.

The article "Photo-responsive hole formation in the monolayer membrane wall of a supramolecular nanotube for quick recovery of encapsulated protein" was retracted in 2024. Reasons: fabricated or falsified images; an official misconduct investigation; misconduct by an author; errors in the images.

**Fig. 6:** (a–c) Scanning electron micrographs of GlcC_18_-GlcGlyAzo-tubes after ultraviolet irradiation for 5 min. Red and blue arrows indicate holes within the monolayer membrane walls made by ultraviolet irradiation and the original holes at the open ends of the tubes, respectively. (d) Schematic representation showing how exposure to ultraviolet light induces *trans*-to-*cis* photoisomerization and dissociation of GlcGlyAzo components from the monolayer membrane wall, leading to the formation of holes.

We hypothesized that the formation of holes in the monolayer membrane of the nanotube would influence the speed of release of compounds encapsulated within the one-dimensional cavity. To examine this hypothesis, we constructed nanotubes within which a model protein, green fluorescent protein (GFP), was encapsulated. The nanotubes were stored in water at pH 6.8, a pH at which GFP is negatively charged (isoelectric point, 4.7–5.1)^29^ and the carboxyl groups on the inner surface of the nanotubes are also negatively charged due to partial deprotonation.^16,17,30^ The release of GFP from the nanotubes into the bulk solution was monitored over time with and without UV irradiation (Fig. 7). Without UV treatment, GFP was found to be slowly released from the open ends of GlcC_18_-GlcAzo-tube and GlcC_18_-GlcGlyAzo-tube, which was attributed to there being no interaction between GFP and the carboxyl groups on the inner surface of the nanotubes; at 24 h after the start of monitoring, the release ratios were only 40–45% (Fig. 7a and b). In contrast, with UV irradiation, hole formation as the result of *trans*-to-*cis* isomerization and subsequent dissociation of the GlcGlyAzo component led to rapid release of GFP from GlcC_18_-GlcGlyAzo-tube; at 1 h after the start of UV irradiation, the release ratio was around 60% (Fig. 7d). These results indicate not only that the original open ends but also the holes that formed in the membrane wall allowed the release of GFP from the nanotubes into the bulk solution. These results also confirm that the holes were sufficiently large for GFP to pass through. Such rapid release of GFP upon UV irradiation was not observed for GlcC_18_-GlcAzo-tube (Fig. 7c), further demonstrating the lack of photoisomerization and dissociation of the GlcAzo component from the monolayer membrane.

The article "Photo-responsive hole formation in the monolayer membrane wall of a supramolecular nanotube for quick recovery of encapsulated protein" was retracted in 2024. Reasons: fabricated or falsified images; an official misconduct investigation; misconduct by an author; errors in the images.

**Fig. 7:** Time dependence of recovery ratios of (a, c) the GlcAzo component of GlcC_18_-GlcAzo-tube and green fluorescent protein (GFP) encapsulated in GlcC_18_-GlcAzo-tube, and (b, d) of the GlcGlyAzo component of GlcC_18_-GlcGlyAzo-tube and GFP encapsulated in GlcC_18_-GlcGlyAzo-tube. Note the different time scales between the upper and middle panels. (e, f) Representative fluorescence micrographs of GFP released from the open end of GlcC_18_-GlcAzo-tube and from the holes in the membrane wall of GlcC_18_-GlcGlyAzo-tube.

Fluorescence microscopy allowed visualization of the release of GFP from the nanotubes (Fig. 7e and f). Two patterns of fluorescence were observed: fluorescence in a straight line, which we attribute to GFP encapsulated in the nanotubes, and fluorescence in clumps, which we attribute to the accumulation of GFP on the outside of the nanotubes after release. The possibility of nonspecific adsorption of GFP on the outer surface of the nanotubes during preparation of the nanotubes encapsulating GFP can be ruled out because the glucose headgroups on the outer surface of the nanotubes were also negatively charged, which would have prevented adsorption of GFP due to electrostatic repulsion.^31^ Thus, GFP existing on the outside of the nanotubes was GFP released from the nanotubes. In the case of GlcC_18_-GlcAzo-tube, fluorescence was observed only along the length and at the ends of the nanotube, indicating that GFP was released only from the original open ends of the nanotube (Fig. 7e). In contrast, in the case of GlcC_18_-GlcGlyAzo-tube, fluorescence was observed along the length and on the outside of the middle part of the nanotube, but not at the ends, indicating that GFP was preferentially released from the holes that formed in the membrane wall rather than from the original open ends of the nanotube (Fig. 7f).

The article "Photo-responsive hole formation in the monolayer membrane wall of a supramolecular nanotube for quick recovery of encapsulated protein" was retracted in 2024. Reasons: fabricated or falsified images; an official misconduct investigation; misconduct by an author; errors in the images.

## Conclusions

A photoresponsive nanotube consisting of a single monolayer membrane was produced by co-assembly in water of a glycolipid and an azobenzene derivative. The azobenzene derivative formed a *J*-type aggregate that was dispersed throughout the glycolipid monolayer membrane. UV irradiation induced *trans*-to-*cis* isomerization of the azobenzene derivative resulting in disassembly of the *J*-type aggregate and dissociation of the azobenzene derivative from the nanotube, which resulted in the formation of many nanometer-scaled holes in the membrane wall. A model protein encapsulated within the nanotubes was rapidly and preferentially released into the bulk solution *via* these holes in the membrane wall compared with that *via* the original two open ends of the nanotube. Thus, the present approach represents a means of recovering guest proteins without exposing them to stimuli that may alter their structure. These findings are expected to be useful for the development of nanocapsules that are able to release substances on demand in response to external stimuli for biological and medical applications.

## Conflicts of interest

There are no conflicts to declare.

## Supplementary Material

NA-004-D2NA00035K-s001
